# Research on the Path of Network Opinion Expression in AI Environment for College Students

This article has been retracted.

**DOI:** 10.1155/2021/4360792

**Published:** 2021-12-06

**Authors:** Yue Zhu, Muhammad Talha

**Affiliations:** ^1^Wuxi City College of Vocational Technology, Jiangsu, Wuxi 214000, China; ^2^Department of Computer Science, Superior University Lahore, Pakistan

## Abstract

Network interaction has evolved into a grouping paradigm as civilization has progressed and artificial intelligence technology has advanced. This network group model has quickly extended communication space, improved communication content, and tailored to the demands of netizens. The fast growth of the network community on campus can assist students in meeting a variety of communication needs and serve as a vital platform for their studies and daily lives. It is investigated how to extract opinion material from comment text. A strategy for extracting opinion attitude words and network opinion characteristic words from a single comment text is offered at a finer level. The development of a semiautonomous domain emotion dictionary generating technique improves the accuracy of opinion and attitude word extraction. This paper proposes a window-constrained Latent Dirichlet Allocation (LDA) topic model that improves the accuracy of extracting network opinion feature words and ensures that network opinion feature words and opinion attitude words are synchronized by using the location information of opinion attitude words. The two-stage opinion leader mining approach and the linear threshold model based on user roles are the subjects of model simulation tests in this study. It is demonstrated that the two-stage opinion leader mining method suggested in this study can greatly reduce the running time while properly finding opinion leaders with stronger leadership by comparing the results with existing models. It also shows that the linear threshold model based on user roles proposed in this paper can effectively limit the total number of active users who are activated multiple times during the information diffusion process by distinguishing the effects of different user roles on the information diffusion process.

## 1. Introduction

With the continuous advancement of Internet technology, people's communication methods on the Internet have also undergone significant changes, from searching for information, reading news, and watching videos to gathering and discussing in groups such as Weibo, QQ, and WeChat [1]. This type of network group disrupts traditional face-to-face gatherings and discussions, allowing everyone to share information in a virtual Internet space, resulting in a diverse public space of discourse and a network of action organizations, which has become the interpersonal and emotional connection of college students. College and university network organizations now span all facets of student life, education, and communication. To some degree, these network groups may facilitate diverse interactions and serve as a vital platform for students' studies and living [2, 3]. However, the Internet community is also influencing their study habits, lifestyle thinking patterns, and overall personality development. College students are fast thinkers and receptive to new ideas. They like expressing their thoughts on national politics, social hotspots, and what they have seen and heard in the Internet community, but they lack reasonable thought and judgement, lack education and experience, and have inadequate perspectives on subjects. When expressing thoughts, it is natural to be influenced by the opinions of others. Additionally, some students lack political awareness, moral awareness, and legal understanding, resulting in the spread of incorrect viewpoints among the online community [4].

In order to gain a better understanding of social network public opinion, it is necessary to grasp the development status and characteristics of social network public opinion, systematically summarize the value form of social network public opinion, and analyze the reasons for the formation of social network public opinion [5]. The use of mobile Internet and smart terminals to create new communication technologies, the media advantages of social media to demonstrate the value of public opinion, netizens' reasonable demands for their own legitimate interests, and government management networks to create a clear and rational cyberspace are all examples of social network public opinion research theories [6, 7]. Any kind of research system structure is related to each other according to certain rules and reveals certain internal laws of the system. The theoretical significance is mainly reflected in the research of this article to promote the construction of the social network public opinion research theoretical system, propose a social network public opinion research mechanism model from the perspective of information ecology, and provide a new research perspective for the research of social network public opinion communication. The practical significance is mainly reflected in the research of this article on the basis of theoretical research to promote the construction of early warning and monitoring mechanisms for the evolution of social network public opinion events, guide relevant public opinion management departments to manage network users, and guide relevant public opinion management departments to manage network user relationships.

The processing process is investigated for text preprocessing, and NLPIR-based comment text segmentation and part-of-speech tagging algorithms are primarily presented. In terms of sentiment dictionary-based opinion and attitude word extraction, the extraction of opinion and attitude words is accomplished by establishing a domain sentiment dictionary. A window-constrained LDA network opinion feature word extraction technique is suggested for extracting feature words of network opinions. The algorithm's efficacy and accuracy are confirmed by several experimental comparisons. The TSRank technique introduced in this work is enhanced by adding clustering to find candidate opinion leaders using the UserRank algorithm, considerably reducing the program's execution time. While the TRank system performs somewhat worse when identifying people with more theoretical user influence capabilities, it performs much better when identifying persons with greater actual user influence capabilities. Simultaneously, when the total number of opinion leaders to be found is modest, the TRank method performs better. As a result, the TSRank method suggested in this work is both valid and accurate. In comparison to the LT, the K-LT model introduced in this article, the linear threshold model URI-LT based on user roles may provide a more accurate interpretation of genuine social networks when modelling the process of information diffusion. As a result, the linear threshold model described in this research is both rational and effective.

## 2. Related Work

There are few foreign literatures on college students' online community and the expression of college students' online opinions [8]. They mainly study the fields related to online community opinions and online opinion leaders. Opinion leaders were initially postulated by Lazarsfeld, and they were mostly in the political field at first, before progressively expanding to other parts of life [9, 10]. It is often assumed that foreign research opinion leaders on the Internet are primarily concerned with identity, traits, and kinds. There is a dearth of study on fundamental notions such as influence and impact, and much less is coupled with college students' ideological indoctrination. Related academics' public views are regarded to be the first type of social public opinion. With the introduction of the Internet, the Internet community's viewpoints have been expressed [11]. Because the Internet's popularity in Western countries predates that in the domestic market, there are also numerous works on the Internet community's opinions, but they tend to focus on applied disciplines, and more are needed to examine the Internet community's opinions and influence from a variety of perspectives.

Considering the dissemination of two distinct types of information with distinct release times and assuming that the content of each message may be unrelated to the content of the other messages, related scholars proposed an information diffusion model in which dual information is simultaneously and dynamically propagated in a complex network, as well as a model of dual information infection propagation [12]. The researchers proposed a public opinion propagation model with an incubation period that is continuously contagious in social networks [13]. Through the analysis of the model, the noninfection balance reaches a local stable state, and the geometric method of ordinary differential equations demonstrates the global stability of the noninfection balance [14]. Related scholars have discussed the role of cognitive beliefs in influencing online users' decision to share online hot events [15]. Cognitively naive participants are more likely to share online hot events than participants with strong cognition. Relevant scholars consider the counterattack mechanism and build a rumor dissemination model in a complex network [16]. They believe that the final state of the rumor dissemination process increases with the increase in self-resistance. Researchers established a dynamic model of network malware spreading on scale-free networks based on the rumor spreading model and proposed a model where exposure-infection-recovery-inoculation states are susceptible, and further improvements were made to increase the time of inoculation [17].

Relevant researchers have presented a microscopic risk diffusion model that forecasts the dynamic spread of network risks and threats from a microprobability viewpoint and gathers the most likely infected border nodes at the moment to withstand network risks and threats [18]. Assuming that the dissemination of public opinion crisis information on social media is a competitive process between true and false information, relevant scholars discussed the dissemination characteristics of crisis information at various stages of dissemination and proposed a competitive model of crisis information dissemination [19]. The researchers quantified the virus's spreading impact in the presence of search engines, as well as the virus's spreading process' stability. They presented a popular feedback model by evaluating the community structure of social networks in order to prevent the virus from spreading. The life cycle hypothesis is used by academics to separate the development of online public opinion into stages [20]. In the process of the evolution of online public opinion, opinions are prone to differentiation, opposition, or gathering, resulting in group polarization phenomena such as online confrontation and online condemnation.

Related academics use the knowledge map approach to separate the subject attributes of the map's entities, extract the topic and time attributes of the map's entities from the Neo4j graph database, and trace the development of public opinion themes using multidimensional feature fusion analysis [21]. Relevant researchers have developed an evolutionary game model to include the strategic interactions between Internet media and local governments into a more accurate model of infectious illness [22]. Simultaneously, in light of anticipated utility theory's limitations in defining the profit and loss of game subjects, they analyzed the implications of various local government guiding tactics on the evolution of public opinion. Researchers proposed a dynamic network model of public opinion development and investigated modelling theories such as the dynamic network model's structure, evolution features, and description methodologies [23]. The relevant researchers outlined the important elements influencing the development of emergent network public opinion by comparing and assessing the performance of the five case events and the similarities and variations in the transmission channel of the network public opinion at each stage [24]. Numerous elements influence the development of online public opinion, and researchers have differing views on this part of study, including the division of evolution into three, four, and six phases, and the law of evolution needs to be carefully clarified by scholars [25].

## 3. Corpus Construction and Knowledge Graph Construction

### 3.1. Corpus Construction

Because network public opinion event propagation and diffusion analysis entails opinion leader mining, knowledge graph visualization, and communication and diffusion analysis, corpus labeling, character encoding, and time slicing are necessary for the network public opinion event corpus.

1. Corpus labeling

Opinion leaders play a pivotal role in the spread of online public opinion. Therefore, for the analysis of the spread and spread of online public opinion events, it is necessary to dig out opinion leaders. In order to verify the effectiveness of opinion leader mining, it is necessary to label the opinion leaders in the real data set. Combining the corpus of online public opinion events and the development law of online public opinion, this article will mark Sina Weibo users who meet the following four aspects as opinion leaders: (1) users who are parties to the event; (2) Sina Weibo is marked as “Big V”; (3) users who forwarded more than 300 events; and (4) official Weibo users such as government, schools, and news media.

(2) Character encoding

This article uses the Neo4j graph database as the platform for storing knowledge graphs. The Neo4j database only supports files in UTF-8 encoding format, so the encoding format of the network public opinion event corpus needs to be uniformly adjusted to UTF-8 encoding.

(3) Time slice

The division of the life cycle of online public opinion is very important for the analysis of the spread and spread of online public opinion. According to the online public opinion life cycle theory, the online public opinion event corpus data is divided by time.

### 3.2. Construction of Knowledge Graph of Internet Public Opinion Events

The network public opinion event knowledge graph belongs to the domain knowledge graph, and the construction of the domain knowledge graph usually adopts top-down construction technology. Firstly, the network public opinion event is modelled on the ontology, and the concepts, entities, attributes, and relationships of the network public opinion event corpus are sorted out. In order to ensure the reliability of the graph, the ontology layer is manually verified; then, knowledge acquisition, entity linking, and elimination are completed in sequence. The quality of network public opinion event knowledge is evaluated.  Figure 1 shows the schematic diagram of constructing the knowledge graph of network public opinion events.

The purpose of knowledge representation and reasoning is to transform the triples of the knowledge graph into computable discrete vectors through the representation of knowledge in the knowledge graph, and then, the completion of the knowledge graph and relational reasoning can be performed through calculations between vectors. This paper proposes an attenuation attention mechanism and embeds it in the graph attention network to form a graph attenuation attention network. Knowledge representation and reasoning are carried out by using a graph attenuation attention network.

## 4. Extraction of Opinion Content in Comments Based on the Topic Model

### 4.1. Analysis of the Opinion Content Extraction Algorithm

Opinion content extraction differs from traditional text content extraction in that it requires the extraction of network opinion feature words, opinion attitude words, and the collocation connection between the two from the comment text, and the quantity of data collected is rather significant. There are several studies now being conducted on the extraction of views and attitudes, most of which are accomplished with the use of emotion dictionaries, and public dictionaries are accessible. This paper proposes to extract the network opinion feature words and their positions using the emotion dictionary method first and then extract the network opinion attitude words using the LDA topic model based on the position of the opinion words, in order to achieve simultaneous extraction of the network opinion feature words and the opinion attitude words to ensure Internet opinion character. The working flow chart of the opinion content extraction algorithm described in this article is shown in Figure 2.

It can be seen from Figure 2 that the entire algorithm receives text content as input and then finally outputs the content of opinions after extracting opinions and attitude words based on the sentiment dictionary and extracting network opinion feature words based on the topic model. Obviously, there are three more critical tasks, namely, text preprocessing, opinion, and attitude word extraction based on sentiment dictionary and network opinion feature word extraction based on the topic model.

Information gain (IG) represents the difference between the quantity of information available when a certain feature item is present and the amount of information available when it is absent. Accordingly, information gain may be viewed as the criticality of the feature item and can be utilized as a criterion for whether or not a feature is kept. The entropy determines how much information is available for categorization. The information gain is equal to the difference between the original entropy of the system and the conditional entropy of the feature item *t*_*k*_, as shown in the following formula:

(1) $$\begin{array}{c} \text{Gain}\left(t_{k}\right)=\left|\text{Entropy}\left(S\right)\right|-\left|\text{Expected}\_\text{Entropy}\left(S_{k}\right)\right|. \end{array}$$

The entropy of *M* categories of documents is defined as follows, where *P*(*C*_*j*_) represents the probability of documents of category *C*_*j*_ appearing in the training set.

(2) $$\begin{array}{c} \text{Entropy}\left(S\right)=-\overset{M-1}{\underset{j=0}{\prod }}\left\{P\left(C_{j}\right)\log\left[P\left(C_{j}\right)\right]\right\}. \end{array}$$

The conditional entropy of the feature item is defined as follows, where *P*(*t*_*k*_) represents the probability that documents with the feature *t*_*k*_ appearing in the training sample.

(3) $$\begin{array}{c} \text{Expected}\_\text{Entropy}\left(S_{k}\right)=-\left[1-P\left(t_{k}\right)\right]•\overset{M-1}{\underset{j=0}{\prod }}\left\{P\left(C_{j}\left|t_{k}\right.\right)\log\left[P\left(C_{j}\left|t_{k}\right.\right)\right]\right\}. \end{array}$$

The final expression of information gain is

(4) $$\begin{array}{c} \text{Gain}\left(t_{k}\right)=-\left[1-P\left(t_{k}\right)\right]•\overset{M-1}{\underset{j=0}{\prod }}\left\{P\left(C_{j}\right)\log\left[P\left(C_{j}\left|t_{k}\right.\right)\right]\right\}+P\left(t_{k}\right)•\overset{M-1}{\underset{j=0}{\prod }}\left\{P\left(C_{j}\left|t_{k}\right.\right)\log\left[1-P\left(C_{j}\left|t_{k}\right.\right)\right]\right\}. \end{array}$$

### 4.2. Text Preprocessing

The language style of comments written by users varies from person to person and does not completely conform to the grammatical rules. In order to ensure the accuracy of the comment content extraction model, preprocessing is required.

Different applications have different processing requirements, and the preprocessing process will be adjusted accordingly. For example, this article preprocesses comment texts, mainly to filter invalid comments and filter out words that do not contribute to the expression of opinions.

Word segmentation and part-of-speech tagging are to find out the Chinese words and their parts of speech (adjectives, nouns, verbs, etc.) in the text. Word segmentation and part-of-speech tagging technologies are quite mature, like NLPIR, which is a widely used word segmentation system. This article is based on the NLPIR word segmentation system and adds it to the NLPIR user dictionary by constructing a dedicated vocabulary word segmentation dictionary in the e-commerce field. Since the priority of the user dictionary is higher than that of the word segmentation system, it can ensure that the proprietary vocabulary is correctly recognized. For example, the high-end and high-grade emotional word “Gao Dashang” that describes things should be recognized as one word instead of multiple words.

### 4.3. Opinion and Attitude Word Extraction Based on Sentiment Dictionary

The process of creating the emotional vocabulary is separated into two phases: the first phase involves the construction of the basic dictionary, and the second phase involves the expansion of the basic lexicon. The extension of the sentiment dictionary is classified as domain and synthetic sentiment word expansion. The emotion dictionary's building process is shown in Figure 3.

The template of the basic dictionary in this article comes from the emotional vocabulary ontology database. By extracting the positive and negative words, the rare and uncommon words are removed. The expansion of the domain words is realized by the operation based on semantic similarity. When preprocessing the review corpus, if a new word that is not included in the basic dictionary appears, the semantic similarity between it and the reference word is calculated, the qualified words are put into the candidate dictionary, and the candidate new words are finally evaluated. The semantic similarity is obtained through the point mutual information operation, which can be used to measure the similarity of two words. The calculation formula is as follows:

(5) $$\begin{array}{c} \text{PMI}\left(x,y\right)=\log\left\{\frac{P\left(x,y\right)}{P\left(x\right)•P\left(-y\right)}\right\}. \end{array}$$

Among them, *P*(*x*, *y*) represents the probability that the words *x* and *y* appear together in a certain type of document, *P*(*x*) represents the probability that the word *x* exists alone in a certain type of document, and *P*(*y*) represents the word *y* in a certain type of document probability of unique existence in the document.

### 4.4. Extraction of Internet Opinion Feature Words Based on the LDA Topic Model

Unsupervised learning is achieved using the Latent Dirichlet Allocation (LDA) model. It is mostly employed in the area of text analysis for calculating text data set similarity, prospective topic mining, and document summary production. It is effectively a three-layer Bayesian network, with one-layer networks for documents, subjects, and words. A bag-of-words model is used to turn text input into computer-calculable word frequency information.

In the LDA model, the known data is the words in the text, each subject is a random combination of words in the vocabulary, and each text is a random variable composed of various subjects, and all of them satisfy multiple items.

(6) $$\begin{array}{c} W\left|\left(Z,\phi \right)\right.=\text{Multinomial}\left(-\phi \right), \end{array}$$

(7) $$\begin{array}{c} Z\left|\theta =-\text{Multinomial}\left(\theta \right)\right.. \end{array}$$

Under the condition of the document *d*_*j*_, the probability of the word *w*_*j*_ is

(8) $$\begin{array}{c} P\left(w_{j}\left|d_{j}\right.\right)=\overset{K-1}{\underset{s=0}{\prod }}\left[P\left(s=z\left|d_{j}\right.\right)•P\left(s=z\left|w_{j}\right.\right)\right]. \end{array}$$

LDA is an unsupervised learning model. You only need to set and optimize the model parameters. There is no need to manually mark the text of the training set, which saves manpower and time and is suitable for large-scale corpus processing. Compared with other topic methods, LDA has stronger generalization ability, is not prone to overfitting problems, and performs well in text information dimensionality reduction and topic information clustering. These advantages make the LDA model very suitable for network opinion feature word extraction. Therefore, this paper uses LDA to extract network opinion feature words.

## 5. Simulation Experiment and Analysis

### 5.1. Opinion Leader Mining Simulation Experiment

#### 5.1.1. Obtain the Opinion Leader Candidate Set

To begin, this article develops a social network graph model in order to determine the number of two-degree neighbours, the number of *K* cores, and the two-degree neighbour aggregation coefficient for each node in the graph. After performing maximum and minimum normalisation on the three attribute values, respectively, the zero value of each attribute is substituted with a nonzero minimum value to enable computation of the fourth attribute. We begin the clustering procedure by selecting the optimal cluster number *K* using the elbow approach. Set 2k20 which is shown in Figure 4, as is the elbow diagram. As seen in Figure 4, the clustering effect is rather strong when *k* = 10.

#### 5.1.2. Possibility of Theoretical User Influence

As seen in Figure 5, the LDA topic model performs best in identifying the most important Top-N opinion leaders when each user's followers have the same impact weight. The LT-a model is totally based on the topology of social networks for the purpose of simulating information dispersion. The LDA topic model is an enhanced PageRank algorithm that can accurately assess a user's efficacy inside a social network structure. As a result, the LDA topic model outperforms the other models in terms of theoretical user impact. Because the UserRank and TRank algorithms are heavily influenced by the user's actual past behavior data, the LT-a topic model performs significantly worse in simulations than the LDA topic model. Although the ClusterRank method only uses social network topology to identify opinion leaders, it only uses the aggregation coefficient and the number of fans to quantify user effect. ClusterRank's low performance on the LT-a model demonstrates that the number of fans is no longer adequate to define users. At the same time, it can be seen from Figure 5 that the performance of the UserRank algorithm is lower than that of the LDA topic model. This shows that the opinion leader mining algorithm proposed in this paper has a better mining effect without clustering to obtain the candidate opinion leader set. The overall performance of the TSRank algorithm is low, because TSRank reduces the accuracy in the process of clustering to obtain candidate opinion leaders.

It can be seen from Figure 6 that when the user influence weight is calculated based on the user's historical behavior data, as the value of *N* increases, the performance of the LDA topic model is still optimal. This is because the LDA theme model calculates user influence and activity based on user previous behavior data, while the UI-LR algorithm generates initial user influence based on user past behavior data. Therefore, the Top-N opinion leaders identified by the LDA topic model are closer to the opinion leaders in real social networks. The overall stability of the TSRank algorithm is better.

#### 5.1.3. Actual User Influence Ability

*C*-value counts how many different users can be affected by the microblogs published or reposted by Top-N opinion leaders of each algorithm in the historical behavior of users. It can be seen from Figure 7 that in terms of *C*-value, the performance of the LDA topic model is better than that of the other four algorithms, indicating that the LDA topic model is more accurate in identifying users with high influence in the history.

### 5.2. Information Dissemination Model Simulation

#### 5.2.1. The Influence of Different Attenuation Factors *б*

On the basis of the LT algorithm, first considering that the user influence weight is affected by the time decay factor, the T-LT model is proposed. We set the initial influence weight of the T-LT algorithm. In order to make the diffusion effect only affected by the attenuation factor and the seed node, this paper uniformly sets the threshold *θ* = 0.5 for each user. Considering that when the attenuation factor *б* is too large, the attenuation effect on the node's influence weight is too large, the influence cannot be effectively accumulated. Therefore, we set the value of *б* to (0, 1.2). With 0.05 as the increment, we study the influence of different *б* values on the diffusion effect.

Figure 8 shows how a single seed node is affected by different attenuation factors. A, B, and C in the figure represent different seed nodes. The horizontal axis represents different attenuation factors. When the attenuation factor is equal to 0, the T-LT model is equivalent to the LT model. The total number of users that the seed node set may affect under the associated temporal attenuation factor is shown on the vertical axis. When the attenuation factor is more than 0, the total number of users impacted by the seed node set swings as a whole, as seen in Figure 8. The topological attributes of nodes A, B, and C are displayed in Table 1 by in-depth study in order to investigate the causes for various shifting patterns.

As seen in Table 1, the A node has a modest number of fans, a long diffusion span, and a low diffusion effectiveness value. It demonstrates that node A has a large number of secondary fans (the spreading breadth minus the number of fans equals the number of secondary fans), and the association between fans and secondary fans is weak, implying that activation requires numerous tries throughout the diffusion process. The state has a very tiny following. When the attenuation factor is minimal, the fans are unaffected during the early stages of dissemination, resulting in a minor change in the overall number of people impacted. When the attenuation factor is increased, the number of fans effectively triggered during the first stage of diffusion decreases, resulting in a significant reduction in the overall number of users impacted. Node B has a high fan count, a low secondary fan count, and a high diffusion effectiveness value, suggesting that there are more connections between fans and secondary fans. Even though the attenuation factor is small, the overall number of affected users is much reduced, implying that more fans need many activation attempts before getting activated throughout the spreading phase. Similarly, it demonstrates that among the fans and second-level fans of node C, the number of users who must be activated numerous times before becoming active is also rather high. Compare the experimental results of LT, T-LT, R-LT, URI-LT, and K-LT.

After separately analyzing the influence of time attenuation factor and user influence weight on information diffusion, this paper proposes the URI-LT algorithm based on LT, considering the time attenuation factor and user influence weight at the same time. We analyze the diffusion effect of the same seed node set on different information diffusion models. Here, we set the threshold *θ* = 0.5 for each user. According to the impact analysis results of different *б* values, the attenuation factor *б* = 0.3 is selected to make the impact of the attenuation factor on information diffusion more obvious. Based on the analysis of the influence of different proportions of opinion leaders, the total number of opinion leaders *N* = 60 is selected.  Table 2 shows the comparison of information diffusion results of different information dissemination models.

According to the records in Table 2 and comparing the results of information diffusion with different information dissemination models, it can be found that when the seed nodes are the same, the information diffusion results predicted by T-LT, URI-LT, and K-LT are all smaller than those of the LT model and R-LT model. The predicted results of LT are not much different from the results of the LT model. This is because the T-LT model effectively filters some nodes that require multiple activations to transform into an activated state through a time decay factor. In a real social network, when a user contacts the same information multiple times without reposting it, the probability that the user will eventually repost the information is extremely small. The T-LT model assumes that a user's influence weight will diminish with time and that users who have been exposed to information for a long period without forwarding it will not be able to properly transition into an active state.

## 6. Conclusion

This paper proposes a method of synchronously extracting the opinion attitude words of a single comment text and the network opinion characteristic words at a fine-grained level. The accuracy of opinion and attitude word extraction is increased by developing a semiautonomous domain emotion dictionary generation approach. A window-constrained LDA topic model is developed, which employs the position information of opinion attitude words to increase the accuracy of network opinion feature word extraction and guarantees that network opinion feature words and opinion attitude words are synchronized. Finally, the substance of comments is extracted from the comment text. For the same seed node, the total number of users that the URI-LT model can affect is smaller than the total number of users that the LT model can affect but substantially more than the total number of users that the K-LT model can affect. It demonstrates that the URI-LT model is very accurate when user roles and temporal attenuation effects are taken into account. Additionally, by comparing the results of R-LT, T-LT, and URI-LT information diffusion, this paper discovers that when the weight of the user's influence is distributed according to the user's role concurrently, the weight of the user's influence is dynamically accumulated according to the time decay factor. This is because, when determining the relative significance of users across user roles, this article restricts the relative relevance of users to the range [1, 2]. However, in real-world social networks, the proportional value of users is much larger. Therefore, the role of user roles in the URI-LT model can be strengthened by adjusting the value range of the relative importance of users. This paper proposes a two-stage framework for mining opinion leaders based on the existing opinion leader mining methods to mine opinion leaders from all network users, which causes high computational complexity. The framework is more effective in reducing computational complexity, but there are still some shortcomings in terms of computational accuracy, and subsequent improvements are needed. At the same time, the linear threshold model proposed in this paper based on the improvement of user roles can effectively show the role of opinion leaders in promoting information dissemination in social networks, but there are still shortcomings in calculating the relative importance between users.

## Figures and Tables

**Figure 1:** Schematic diagram of the construction of the knowledge graph of Internet public opinion events.

**Figure 2:** Work flow chart of the opinion content extraction algorithm.

**Figure 3:** The construction process of sentiment dictionary.

**Figure 4:** Elbow diagram.

**Figure 5:** LT-a model simulation comparison results.

**Figure 6:** LT-b model simulation comparison results.

**Figure 7:** *C*-value comparison result.

**Figure 8:** A single seed node is affected by different attenuation factors.

**Table 1:** Topological properties of nodes A, B, and C.

Node	Spread	Diffusion depth	Diffusion effectiveness	Number of fans
A	1220	6	0.0001	140
B	650	5	0.0002	506
C	210	3	0.0001	201

**Table 2:** Comparison of information diffusion results of different information dissemination models.

Number of seed nodes	K_LT	T_LT	R_LT	URI-LT	LT
5	121	1100	1189	1122	1201
10	1990	2890	3009	2986	3011
15	3001	4001	4054	4001	4055
20	4200	4890	4899	4887	4974
25	5129	5720	5776	5701	5691

## Data Availability

Data are available upon request.
